# An Analysis of the Effect of Noninvasive Positive Pressure Ventilation on Patients with Respiratory Failure Complicated by Diabetes Mellitus

This article has been retracted.

**DOI:** 10.1155/2022/3597200

**Published:** 2022-10-14

**Authors:** Jia-an Sun, Xiaoman Wang, Ying Liu, Chang Liu

**Affiliations:** Department of Emergency, Zhengzhou Central Hospital Affiliated to Zhengzhou University, Zhengzhou 450000, China

## Abstract

**Objective:**

To observe the clinical effectiveness of noninvasive positive pressure ventilation in patients with respiratory failure complicated by diabetes.

**Methods:**

From May 2021 to May 2022, 90 patients with respiratory failure complicated by diabetes treated in our hospital were recruited and randomly assigned to receive either medication (control group) or noninvasive positive pressure ventilation (study group), with 45 patients in each group. The clinical endpoint was therapeutic outcomes.

**Results:**

Noninvasive positive pressure ventilation resulted in significantly lower Self-Rating Anxiety Scale (SAS) and Self-Rating Depression Scale (SDS) scores versus medications (*P* < 0.05). Patients with noninvasive positive pressure ventilation showed better pulmonary function indices versus those with medications (*P* > 0.05). There was no significant difference in arterial oxygen (PaO_2_), carbon dioxide partial pressure (PaCO_2_), and arterial oxygen pressure/inspired fraction of O_2_ (PaO_2_/FiO_2_) between the two groups prior to the intervention (*P* > 0.05). However, patients in the study group had significantly elevated PaO_2_ and PaO_2_/FiO_2_ and lower PaCO_2_ levels than those in the control group (*P* < 0.05). Following the intervention, noninvasive positive pressure ventilation resulted in significantly lower inflammatory factor levels versus medications (*P* > 0.05). After the intervention, markedly better glucose control was observed in the study group versus the control group (*P* < 0.05). The incidence of complications in the control group was 2.38%, which was significantly lower than that of the control group (16.67) (*P* < 0.05).

**Conclusion:**

Noninvasive positive pressure ventilation effectively suppresses the inflammatory response, improves the blood gas analysis index, and eliminates the negative emotions of patients, thereby maintaining hemodynamic stability and improving clinical efficacy with a better safety profile. Further studies are recommended prior to clinical promotion.

## 1. Introduction

Chronic obstructive pulmonary disease (COPD) results in a high risk of respiratory failure, and given the decreased immunity of the body with age and physiologic changes related to breathing, COPD features a high prevalence among the elder population and compromises their respiratory function. Moreover, long-term respiratory insufficiency may result in chronic illnesses such as diabetes, and untimely or improper management of the disease is associated with a high risk of disease progression [1, 2]. Diabetes occurs due to the insufficient secretion or use of insulin in the human body. Insulin is a hormone that regulates blood sugar. Hyperglycemia or elevated blood sugar is a common consequence of uncontrolled insulin, which is associated with potential neurological and vascular damage.

Multiple therapeutic approaches such as low-flow oxygen inhalation and atomization therapy have been previously adopted for the management of respiratory insufficiency aggravated by diabetes. However, their efficacy remains much to be desired [3, 4]. In traditional Chinese medicine, diabetes is caused by external factors such as lack of congenital endowment, emotional disorders, overwork, improper diet, and preference for fatty, sweet, and greasy foods, and TCM treatment for diabetes is mainly performed based on the characteristics of patients' symptoms. The combination of Chinese and Western medicine may be the future direction of treatment research.

With the advancement of medical technology, mechanical ventilation has made substantial progress in the treatment of severe respiratory failure and has shown significant therapeutic outcomes [5, 6]. Noninvasive positive pressure ventilation obviates the need to establish an artificial airway. It connects the patient's respiratory airway to the ventilator with the assistance of a nasal cannula or mask, without compromising swallowing function, coughing up sputum, or eating, thus reducing the risk of airway and lung infections and other related complications associated with invasive ventilation (tracheal intubation or tracheotomy). Thus, it is widely used in the clinical treatment of acute COPD exacerbations and acute cardiogenic pulmonary edema. To this end, this study was undertaken to observe the clinical effectiveness of noninvasive positive pressure ventilation in patients with respiratory failure complicated by diabetes.

## 2. Data and Methods

### 2.1. General Data

From May 2021 to May 2022, 90 patients with respiratory failure complicated by diabetes treated in our hospital were recruited and randomly assigned to receive either medication (control group) or noninvasive positive pressure ventilation (study group), with 45 patients in each group. The control group contained 23 males and 22 females, aged 65-84 (69.53 ± 6.78) years, disease duration of 2-9 (6.29 ± 1.43) years, and a body mass index (BMI) of 19-29 (23.73 ± 1.38) kg/m^2^. In the study group, there were 29 males and 16 females, aged 66-85 (69.62 ± 6.85) years, disease duration of 3-10 (6.35 ± 1.48) years, and a BMI of 20-28 (23.82 ± 1.34) kg/m^2^. The patient characteristics between the two groups were comparable (*P* > 0.05).

#### 2.1.1. Random Method

The randomization was carried out using an online web-based randomization tool (freely available at http://www.randomizer.org/). For concealment of allocation, the randomization procedure and assignment were managed by an independent research assistant who was not involved in the screening or evaluation of the participants.

#### 2.1.2. Sample Size Estimation

The original sample size calculation estimated that 40 patients in each group would be needed to detect a 3-point difference between groups in a 2-sided significance test with a power of 0.8 and an alpha error level of 0.05.

#### 2.1.3. Ethical Considerations

The study protocol and all amendments were approved by the appropriate ethics committee at each centre. The study was done in accordance with the protocol, its amendments, and standards of clinical practice. All participants provided written informed consent before enrolment (Ethics No. HU-YU20200103).

#### 2.1.4. Inclusion and Exclusion Criteria

Inclusion criteria (all patients who met the following criteria were included in this study) are the following:

- Patients who had confirmed respiratory failure by clinical examination
- With complete medical history
- With high compliance

Exclusion criteria are the following:

- With neurological disorders
- With insufficiency of important organs
- With abnormal coagulation function
- With immune system disorders, systemic infections, or organic brain diseases

### 2.2. Methods

After admission, the control group received targeted drug treatment, including anti-infection, correction of electrolyte imbalance, nutritional support, blood gas analysis, and ECG monitoring. The study group adopted noninvasive positive pressure ventilation assistance. (a) The oxygen tube was connected to the side port of the mask, and a noninvasive ventilator was connected; (b) the breathing rate was reduced to S/T (lower than the respiratory rate selected by the researcher). In the early stage of the treatment, the initial pressure was set to 1.5 cm H_2_O (1 cm H_2_O is 0.098 kPa), and the inspiratory pressure was set to 4 cm H_2_O, gradually adjusting to 6 cm H_2_O according to the patient's state of health; the respiratory rate was maintained at 25 times per minute, and the oxygen flow was set to 8-12 mL/kg. The patient's physical signs were continuously monitored during treatment, including heart rate, blood pressure, and respiratory rate. The breathing rate was maintained at 20 times per minute, and the inspired oxygen concentration was maintained within 30%. A support pressure of 10 cm H_2_O may be applied externally.

#### 2.2.1. TCM Adjuvant Therapy

All patients received TCM decoction. The ingredients of the decoction include 30 g of gypsum and yam each, 15 g of Trichosandra, 15 g of astragalus, 10 g of dodder, 10 g of Poria cocos, 10 g of Anemarrhena, 5 g of dried radix rehmanniae, 5 g of Ophiopogon japonicus, and 5 g of Scrophulariaceae, which were decocted with water and administered once daily, with a half dose administered in the morning and a half in the evening.

### 2.3. Observational Indices

#### 2.3.1. Psychological Status

The Self-Rating Anxiety Scale (SAS) and Self-Rating Depression Scale (SDS) were used to assess the patient's psychological status before and after the intervention. According to the scale, there are 20 items and a 4-level scoring method. A total score of SAS > 50 and SDS > 50 indicate anxiety and depression.

#### 2.3.2. Pulmonary Function Indices

Before and after the intervention, the forced vital capacity (FVC), forced expiratory volume in one second (FEV1), FEV1/FVC, maximum voluntary ventilation (MVV), and maximum carboxylation capacity (VCmax) of the patients were assessed.

#### 2.3.3. Indices of Arterial Blood Gases

Arterial blood gases were measured before and after the intervention to determine the arterial oxygen (PaO_2_), carbon dioxide partial pressure (PaCO_2_), arterial oxygen pressure/inspired fraction of O_2_ (PaO_2_/FiO_2_), and the oxygenation index.

#### 2.3.4. Inflammatory Factors

5 mL of venous blood was collected from the two groups before and after the intervention and centrifuged at 3000 r/min to obtain the serum. The levels of procalcitonin (PCT) and C-reactive protein (CRP) were measured using the enzyme-linked immunosorbent assay.

#### 2.3.5. Blood Glucose Control

Fasting blood glucose and glycosylated hemoglobin levels were measured before and after the intervention. Between the two groups, complications such as respiratory muscle weakness, ventilator-associated pneumonia, and acute pulmonary edema were recorded.

### 2.4. Statistical Analysis

The mean difference between the two groups was tested using Student's *t*-test for normally distributed variables and the Mann–Whitney *U* test for nonnormal variables. The data were analyzed with the software SPSS 20.0. The count data were expressed as “*n* (%)” and analyzed using the chi-square test. The measurement data were expressed as mean ± standard deviation (“$\bar{x}\pm s$”), and independent *t*-tests were used for comparisons between groups and paired *t*-tests for comparisons within groups. *P* < 0.05 indicates that the difference is statistically significant.

## 3. Results

### 3.1. SAS and SDS Scores

SAS and SDS scores did not differ significantly between the two groups prior to the intervention (*P* > 0.05). Noninvasive positive pressure ventilation resulted in significantly lower SAS and SDS scores versus medications (*P* < 0.05) (Table 1).

### 3.2. Pulmonary Function Indices

Patients with noninvasive positive pressure ventilation showed better pulmonary function indices versus those with medications (*P* > 0.05) (Table 2).

### 3.3. Arterial Blood Gas Indices

There was no significant difference in PaO_2_, PaCO_2_, and PaO_2_/FiO_2_ between the two groups prior to the intervention (*P* > 0.05). However, patients in the study group had significantly elevated PaO_2_ and PaO_2_/FiO_2_ and lower PaCO_2_ levels than those in the control group (*P* < 0.05) (Table 3).

### 3.4. Inflammatory Factors

There was no significant difference in the levels of inflammatory factors between the two groups prior to the intervention (*P* > 0.05). Following the intervention, noninvasive positive pressure ventilation resulted in significantly lower inflammatory factor levels versus medications (*P* > 0.05) (Table 4).

### 3.5. Blood Glucose Control

After the intervention, markedly better glucose control was observed in the study group versus the control group (*P* < 0.05) (Table 5).

### 3.6. Incidence of Complications

The incidence of complications in the control group was 2.38, which was significantly lower than that of the control group (16.67) (*P* < 0.05) Table 6.

## 4. Discussion

COPD is characterized by persistent respiratory symptoms and significant airflow limitations [7, 8]. COPD is a complex disorder with chronic inflammation in the airways, oxidative stress, and an imbalance between proteases and antiproteases. Stable COPD is associated with relatively mild symptoms such as chronic coughing and shortness of breath. Acute lung infection may cause an acute attack by increasing airway blockage, inducing respiratory failure, and resulting in acidosis, resulting in a poor prognosis [8]. Hence, timely and effective treatment measures for COPD are essential to enhance patient prognosis.

At this stage, the clinical treatment measures for COPD complicated with severe respiratory failure primarily include antispasmodic and asthmatic medications, correction of internal environment disturbances, and nutritional support. However, their efficacy remains inconsistent across all patients, especially those with critical illnesses such as diabetes or heart disease. Research has also indicated supplements with ventilation to correct hypoxia and hypercapnia [9]. Additionally, the reduction in oxygen content in the body compromises the normal metabolism, resulting in endocrine metabolism disorders and abnormal secretion of insulin [10]. As a result, patients with respiratory failure and diabetes are more predisposed to develop insulin resistance. It has been reported that respiratory failure and insulin resistance have a dialectical relationship of mutual influence and interaction [9, 11–14]: Hypoxia and hypoxemia caused by chronic respiratory failure impair the function of islet *β*-cells, leading to the abnormal release of insulin release.

Chronic hypoxia in respiratory failure may result in the imbalance between the thalamus, pituitary, and adrenal cortex, followed by a massive secretion of adrenocorticotropic hormone and interfered glucose metabolism, resulting in elevated blood glucose levels. Hypoxia causes compromised efficiency of insulin binding to target cells.

Patients with diabetes are more susceptible to pulmonary infection and airway mucosal congestion, and ciliary movement impairment since airflow limitation exacerbates respiratory failure and complicates the treatment, which necessitates the timely intervention of ventilation measures.

Noninvasive ventilation can effectively correct hypoxia, reduce CO_2_ retention, promote the ability of pancreatic *β*-cells to return to their original function, enhance the metabolism of carbohydrates, and restore blood sugar to a normal level. It provides significant therapeutic benefits for cases of hypoxia and insulin resistance caused by respiratory failure. In the present study, there were no significant changes between the two groups in terms of psychological state ratings, pulmonary function indexes, arterial blood gas indexes, inflammatory factor levels, fasting blood glucose levels, and glycosylated hemoglobin levels before the intervention (*P* > 0.05). Noninvasive positive pressure ventilation resulted in better outcomes in terms of the above indices versus medications (*P* < 0.05), suggesting that this method can be used to effectively improve the arterial blood gas index and effectively mitigate the inflammatory response of the body. The reason may be that timely ventilation clears secretions of the respiratory tract and bronchi, enhances partial pressure of oxygen in the body while dredging the trachea, corrects hypoxemia, improves breathing conditions, and promotes the recovery of arterial blood gas indices. Moreover, ventilation drains sputum, improves respiratory dysfunction, and reduces respiratory muscle fatigue, thereby enhancing tissue oxygen supply, acid-base balance disorders, and compensation for water and electrolyte imbalances. Several studies have shown that noninvasive ventilation could improve gas exchange, correct hypoxemia, control hypercapnia, and improve cardiac function. At this stage, anaerobic glycolysis is converted to aerobic oxidation, which increases glucose metabolism, decreases liver glycogen disintegration and release, and raises blood sugar levels. The vagus nerve and cardiopulmonary receptors are activated to promote insulin sensitivity [15–17].

Furthermore, the present study revealed a lower incidence of complications in the study group (2.38%) versus the control group (16.67%), indicating a high safety profile. It has been stated that noninvasive positive pressure ventilation should be used as early as possible to dilate the pulmonary blood vessels of patients, thereby maintaining pulmonary functional residual capacity, reducing intrapulmonary shunts, improving pulmonary ventilation, decreasing respiratory failure symptoms, reducing inflammation caused by hypoxia, and accelerating recovery [18]. The reason may be that noninvasive positive pressure ventilation is a form of artificial ventilation assisted by a nasal mask that connects the ventilator to the patient, with the ventilator providing positive pressure support [19]. When this positive pressure is reduced or withdrawn, the whole chest and lungs rebound, and gas is exhaled, which allows ventilation equivalent to physiological breathing and negative pressure ventilation. However, the damage to the lungs of elderly patients with diabetes mellitus combined with severe respiratory failure is difficult to recover by the mechanism of body self-regulation, and this damage is nonpathological damage that compromises the treatment efficiency of pharmacological treatment [20, 21].

Noninvasive positive pressure ventilation effectively suppresses the inflammatory response, improves the blood gas analysis index, and eliminates the negative emotions of patients, thereby maintaining hemodynamic stability and improving clinical efficacy with a better safety profile. Further studies are recommended prior to clinical promotion. However, it is worth noting that the operation of noninvasive positive pressure ventilation differs from invasive ventilation in that more emphasis is placed on the standardization of the operation and adequate communication with the patient. The standard of operation is directly related to the effectiveness of noninvasive positive pressure ventilation [22–24].

The present study has the following limitations: (1) the small sample size in this trial failed to objectively evaluate the significant differences between the two groups. (2) This study used more subjective efficacy assessment criteria, and the subjective perceptions of individuals differed greatly, resulting in difficulties in providing an absolutely objective and accurate description of the ratings on the scale. (3) The follow-up period after treatment in this trial was short, which failed to observe the long-term treatment effect.

In conclusion, noninvasive positive pressure ventilation effectively suppresses the inflammatory response, improves the blood gas analysis index, and eliminates the negative emotions of patients, thereby maintaining hemodynamic stability and improving clinical efficacy with a better safety profile. Further studies are recommended prior to clinical promotion.

## Figures and Tables

**Table 1:** SAS and SDS scores ($\bar{x}\pm s$).

Group	Cases	SAS score		SDS score	
		Before intervention	After intervention	Before intervention	After intervention
Control group	45	59.32 ± 4.53	54.32 ± 5.67	59.84 ± 4.35	55.43 ± 6.22
Study group	45	59.35 ± 4.34	48.13 ± 5.16	61.03 ± 4.53	49.86 ± 4.22
*t* value		0.396	6.985	0.353	5.344
*P* value		0.756	≤0.001	0.721	≤0.001

**Table 2:** Pulmonary function indices ($\bar{x}\pm s$, *n* = 45).

Group	FVC (L)		FEV1 (L)		FEV1/FVC		VCmax (L)		MVV (L/min)	
	Before intervention (B.I)	After intervention (A.I)	B.I	A.I	B.I	A.I	B.I	A.I	B.I	A.I
Control group	3.21 ± 0.68	3.45 ± 0.71	2.92 ± 0.42	3.21 ± 0.45	75.27 ± 7.55	80.01 ± 8.46	3.31 ± 0.48	3.63 ± 0.52	79.03 ± 11.02	85.22 ± 11.96
Study group	3.42 ± 0.78	5.51 ± 0.71	2.94 ± 0.45	5.31 ± 0.48	75.03 ± 8.26	90.16 ± 8.82	3.33 ± 0.41	5.71 ± 0.47	79.76 ± 11.01	96.33 ± 15.02
*t*	0.21	13.08	0.19	7.61	0.32	8.36	0.12	7.72	0.33	11.36
*P*	0.82	≤0.01	0.91	≤0.01	0.86	≤0.01	0.91	0.00	0.77	≤0.01

**Table 3:** Arterial blood gas indices ($\bar{x}\pm s$, *n* = 45).

Group	PaO_2_ (mmHg)		PaCO_2_ (mmHg)		PaO_2_/FiO_2_ (mmHg)	
	Before intervention	After intervention	Before intervention	After intervention	Before intervention	After intervention
Control group	51.63 ± 7.66	82.23 ± 6.59	60.03 ± 5.72	42.48 ± 5.13	131.68 ± 8.59	186.77 ± 10.24
Study group	50.47 ± 7.38	90.57 ± 5.62	59.32 ± 5.57	31.37 ± 4.65	130.25 ± 8.35	250.11 ± 12.36
*P* value	0.748	6.602	0.609	11.001	0.818	27.054
*t* value	0.228	0.000	0.272	0.000	0.208	0.000

**Table 4:** Inflammatory factors ($\bar{x}\pm s$).

Group	PCT (*μ*g/L)		CRP (mg/L)	
	Before intervention	After intervention	Before intervention	After intervention
Control group (*n* = 45)	1.23 ± 0.21	0.75 ± 0.16	84.36 ± 6.48	70.54 ± 5.29
Study group (*n* = 45)	1.19 ± 0.26	0.42 ± 0.11	84.45 ± 6.57	62.37 ± 4.57
*t*	0.656	9.309	0.053	6.401
*P*	0.515	≤0.001	0.958	≤0.001

**Table 5:** Blood glucose control effects ($\bar{x}\pm s$).

Group	Glucose level fasting (mmol/L)		Glycated hemoglobin (%)	
	Before intervention	After intervention	Before intervention	After intervention
Study group (*n* = 45)	12.13 ± 0.57	7.26 ± 1.45^ab^	6.21 ± 1.33	5.06 ± 1.95^ab^
Control group (*n* = 45)	11.64 ± 0.76	9.92 ± 1.34^a^	6.46 ± 1.27	8.53 ± 1.77^a^

Note: ^a^compared with after intervention, *P* < 0.05; ^b^compared with the control group, *P* < 0.05.

**Table 6:** Comparison of the incidence of complications among the two groups (*n* (%)).

Group	ICU care	Ventilator-associated pneumonia	Acute pulmonary edema	Overall incidence
Control group	3 (7.14)	2 (4.76)	2 (4.76)	7 (16.67)
Study group	0 (0.00)	0 (0.00)	1 (2.38)	1 (2.38)
*X* ^2^				3.943
*P*				0.018

## Data Availability

No data were used to support this study.
